# Exploring the Path of Enhancing Ideological and Political Education in Universities in the Era of Big Data

**DOI:** 10.1155/2022/2288321

**Published:** 2022-08-31

**Authors:** Nana Shao, He Hu

**Affiliations:** ^1^School of Marxism, Hainan Medical University, Hainan, Haikou 571199, China; ^2^School of Marxism, Qiongtai Normal University, Hainan, Haikou 570204, China; ^3^Hainan Integrated Moral Education Research Base for College, Middle School and Children, Hainan, Haikou 570204, China

## Abstract

The emergence of the big data era has drastically altered people's lives and perceptions. One needs a thorough understanding of the topic to effectively apply big data's benefits to the ideological and political education work that colleges and universities carry out. By doing so, the advantages of big data can be better exploited and integrated into the educational process, enhancing the work's overall quality. To enhance the path of ideological and political education in colleges and universities, it is necessary to change according to the matter, advance according to the time, and make new changes according to the situation, and therefore, it is important to actively explore the path of ideological and political education in colleges and universities under the times. In this study, we research and analyze the opportunities and challenges facing the ideological and political education of universities in the era of big data, reexamine the subjective and objective environment in which the ideological and political education of universities is located, and explore the innovative development path of the ideological and political education of universities in the new environment. We will also encourage the innovative growth of ideological and political work in four areas, such as cultivating big data thinking innovation, working method innovation, working carrier innovation, and ideological work team construction, and conduct a ranking analysis on the significance of the exploration variables to improve the path of ideological work. The importance score measures the value of features in the construction of the ascending decision in the model, so the XGBoost algorithm is used to sort and analyze the significance of exploring variables to enhance the political and ideological work trajectory. The analysis of the experimental results shows that the innovation of working methods has greatly enhanced the conditions for carrying out ideological and political education in the new environment and has far-reaching implications and important significance for the innovation of ideological and political education in universities.

## 1. Introduction

Talent is one of the factors essential to the development of a country, and the cultivation of excellent people requires a decent education. Universities should now prioritize developing talent and creating a strong educational framework so that education can keep up with the trends and produce breakthroughs and innovations. The coming of age of big data has given education a great opportunity [1, 2]. To fully exploit the benefits of big data, universities should develop a big data platform using network information technology. Education's implementation could be done more effectively [3].

Big data's distinctive properties of volume, speed, diversity, and value offer new support and conditions for colleges and universities to innovate in their delivery of political and ideological education within the perspective of the modern world [4]. By collecting a large amount of data related to students, such as personal information on students' families, career planning, grades in various subjects and behavioral information on classroom attendance, social practice, and on-campus and off-campus activities, universities can establish a comprehensive and rich database of ideological and political education resources in talent training and student management services, providing a massive information base for later data analysis. Big data collection and access speed are quick, and it can be used by sensors, the Internet, and other electronic devices and network tools to record students' behavior in real time, *n* order to make ideological and political education more timely and to provide convenient circumstances; big data record structured and unstructured diverse data of students, realizing complete diversity of data on the premise that the amount of completed data is large enough, and all kinds of information are interrelated, supplemented, and modified to ensure the accuracy of future predictions [5, 6]. The attention, tracking, analysis, and processing of big data on education subjects throughout the whole process can help to grasp the comprehensive and dynamic situation of education subjects and carry out continuous follow-up processing, so that educators can accurately and deeply understand the behavior and status of education subjects. The research on big data predicts the possible situation of the education target and takes corresponding educational guidance and helps support, which plays an important role in improving the effectiveness of ideological and political education in universities [7]. Politicians who engage in ideological and political activity using network platforms and information technology have additional challenges, particularly in the following areas: (1) ideological and political efforts receiving insufficient consideration in the big data era. All colleges currently choose their own network platform as a conduit for outside exposure and network political ideas. However, problems such as low levels of human interaction, a lack of resources, a lack of connectivity, and inadequate communication usually appear while developing political and ideological education on the Internet. For engaging in political and ideological teaching activities online, there is a lack of long-term mechanisms and system designs, and institutions frequently place more emphasis on publicity and promotion than education and guiding [8, 9]. (2) The psychological growth of college students is likely to be negatively impacted by moral wrongdoing in the online community. The popularity of the network makes college students susceptible to the effect of all forms of network information, and the virtual nature of the network environment is likely to result in some self-indulgence and disconnection from the realistic way of life during network engagement. Some college students, who have sick psychology, estranged interpersonal communication, and misbehavior, minimize to some extent the influence of political and ideological education work [10, 11]. (3) Network ideological and political platform development needs to be reinforced, and it is urgently necessary to train ideological and political employees in data management. As a result of the growth of network big data, political and ideological educators from the traditional educational model of classroom instruction, one-on-one talks, class meetings, and group meetings to the various development of network education techniques are confronting new obstacles [12].

Colleges and universities have natural advantages in the areas of subject, object, and carrier of teaching in the big data era, which is the area of higher education talent cultivation. As a result, an increasing number of scholars are studying the interactions that arise naturally in higher education institutions between big data and political and ideological education. Big data are being used more and more to teach concepts and politics in college and university courses [13]. Many colleges and universities have looked into the innovative development of political and ideological education in the big data era, as well as real-world applications based on big data in student network behavior, on-campus learning and living behavior, political and ideological theory class teaching, and extracurricular practice. In contrast to the traditional political and ideological education, big data in digital technology simultaneously introduce new methods, challenge conventional wisdom, modify the new approach to learning about the world, alter how people behave in it, and significantly enhance the conditions for political and ideological education in the context of the modern world. A foundation was built for the creation of the work practice of political and ideological instruction. It significantly affects and has a broad impact on the development of political and ideological education at universities [14].

The idea of its education, which is substantially out of date, is one of the key factors preventing the growth of educational institutions today teaching political and ideological ideas. The problem is that teachers do not logically combine big data with classroom teaching during the teaching process, and the cognition of education still focuses on textbook teaching, which does not produce good teaching effects [15]. As we all know, universities primarily view classroom learning as an important method to improve students' ideology and politics. Therefore, educators should integrate big data into their lessons to help students better grasp ideology and politics. Therefore, teachers should combine teaching with big data, use big data to let students watch some typical figures in society, and deliver some positive messages to students through online information, to help students better understand ideology and politics [16, 17].

In the age of big data, many crucial judgments will not be relied on people's firsthand knowledge or intuitive summaries, but rather on data analysis to draw conclusions. Universities can leverage this particular characteristic of big data to develop specialized data and information platforms that can track progress in the field of political and ideological education [18]. Teachers will be able to fully create individual teaching qualities, stay current on students' views and ideological dynamics, and increase the relevance of education in politics and ideology after evaluating the vast amounts of data [19, 20]. In this study, we will conduct a thorough analysis and discussion of big data, as well as the difficulties and potential paths for innovation faced by universities. We will also encourage the innovative growth of ideological and political work in four areas, including the development of big data thinking innovation, working method innovation, working carrier innovation, and ideological work team construction. Additionally, we use the XGBoost algorithm to conduct a ranking analysis of the significance of the exploration factors to enhance the political and ideological curriculum at universities in the hopes that our efforts will be helpful. The experimental results show that the innovation of working methods has greatly improved the conditions of ideological and political education under the new environment and has far-reaching influence and important significance to the innovation of ideological and political education in colleges and universities.

## 2. Related Works

Zhang [21] focused on the relationships between schools, teachers, and students while taking into account the new circumstances and demands of the big data era. He put forth important concepts for the modernization of education in politics and ideology among college students and took into consideration certain tactics and methods for the ongoing application of the ideology and political education in the big data age. In the age of big data, Li [22] proposed that college students construct proper concepts, improve informational skills, create work processes and methodologies, and support the growth of education on ideologies and politics in colleges and universities. Wang and Zhang [23] proposed an innovation in thinking, mode of supervision, and educational mode of thought by concentrating on ideological and political education workers to increase data awareness, improve thinking, and fully grasp big data analysis techniques. By peering into the ideological and political education of the law to prepare for the era of big data, the quality of ideological and political education is improved and the level of education is enhanced. Xia [24] developed a big data artificial intelligence model for managing university ideological and political teaching that is an improvement above the conventional algorithm. Methods for incorporating machine learning into courses on politics and ideologies were presented by Li and Mao [25]. They looked into the political and ideological underpinnings of schooling using the machine learning decision tree algorithm as an example. To assess the outcomes of students who received instruction using our method, the next step is to develop a questionnaire from the perspectives of learning attitude, learning influence, and learning effect. Their research boosted interdisciplinary study and made it simpler for students to understand computer science courses in machine learning, which helped students who majored in both computer science and ideological and political education.

## 3. Modeling Methods and Exploring Talk

### 3.1. XGBoost Algorithm Introduction

The XGBoost algorithm's [26] concept is to continuously add trees and split features to create a tree, and each time a new number is added, it gains a new function to fit the leftovers from the previous forecast [27, 28].  Figure 1 illustrates the main principles of the XGBoost algorithm's operation.

For one of the integrated methods, the mathematical model of the XGBoost algorithm can be represented as follows:

(1) $$\begin{array}{c} {\hat{y}}_{i}=\sum_{k=1}^{K}f\left(x_{i}\right), \end{array}$$

where *K* is the total number of classifiers, *f*(*x*) denotes the *Kth* classifier, ${\hat{y}}_{i}$ denotes the predicted outcome for sample *x*_*i*_ after integrating *K* classifiers, and the loss function is expressed as follows:

(2) $$\begin{array}{c} \text{obj}\left(\theta \right)=\sum_{i=1}^{n}l\left(y_{i},{\hat{y}}_{i}\right)+\sum_{k-1}^{K}\Omega \left(f_{k}\right), \end{array}$$

where $l\left(y_{i},{\hat{y}}_{i}\right)$ is the training error for sample *x*_*i*_, Ω(*f*_*k*_) denotes the regular term for the *kth* tree, Ω(*f*_*k*_)=*γT*+1/2‖*W*‖^2^, and Ω is the complexity of the control model for the penalty term. It also makes *W* smoother and thus avoids overfitting [29]. The optimal parameter *P*^*∗*^ is obtained by minimizing the canonical loss function Ω(*f*_*k*_), which in turn leads to Ω(*f*_*k*_) model *f*^*∗*^(*x*) that is both simple and accurate, and can be expressed as follows:

(3) $$\begin{array}{c} P^{*}=\arg\max\psi \left(x\right). \end{array}$$

Obviously, the solution to *f*^*∗*^(*x*) cannot be calculated directly, so this study considers the optimization method. *f*(*x*) is a decision tree model, given that the weight *W* and tree structure *q* can determine a decision tree, and the tree structure *q* is actually the problem of dividing the split nodes, so it can be translated into the problem of finding the optimal weight W and dividing the split nodes. The specific calculation steps are as follows:

(4) $$\begin{array}{c} y_{i}^{\left(0\right)}=0,\\ y_{1}^{\left(1\right)}=y_{1}^{\left(0\right)}+f_{1}\left(x\right),\\ \ldots ,\\ y_{1}^{\left(t\right)}=\sum_{k=1}^{t}f_{k}\left(x_{1}\right)\\ =y_{1}^{\left(t-1\right)}+f_{t}\left(x\right). \end{array}$$

The approximate objective function is determined in this situation using the Taylor expansion:

(5) $$\begin{array}{c} {\text{obj}}^{t}\left(\theta \right)=\sum_{j=1}^{\gamma }\left\{g_{1}f_{t}\left(x_{1}\right)+\frac{1}{2}h_{t}f_{t}\left(x_{1}\right)\right\}+\gamma T+\frac{1}{2}\lambda T\sum_{j=1}^{T}W_{j}^{2}. \end{array}$$

Since ∑_*j*=1_^*γ*^{*g*_1_*f*_*t*_(*x*_1_)+1/2*h*_*t*_*f*_1_(*x*_1_)} can be thought of as the total of the scores from each sample's score correlation function at the leaf node of the *tth* tree, it can be represented from the leaf node of the *tth* tree:

(6) $$\begin{array}{c} {\text{obj}}^{t}\left(\theta \right)=\sum_{j=1}^{\gamma }\left\{g_{1}f_{t}\left(x_{1}\right)+\frac{1}{2}\sum \left(h_{t}+\lambda \right)W_{j}^{2}\right\}+\gamma T. \end{array}$$

Let

(7) $$\begin{array}{c} G_{1}=\sum g_{1},\\ H_{j}=\sum h_{1}. \end{array}$$

Bringing in the above equation *W*_*j*_, solving for the partial derivative, and then making the derivative function equal to 0, the following equation can be obtained:

(8) $$\begin{array}{c} G_{1}+\left(H_{j}+\lambda \right)W_{j}=0. \end{array}$$

It is obtained that *W*_*j*_^*∗*^=−*G*_*j*_/*H*_*j*_+*λ*.

So, the optimal solution of the objective function is as follows:

(9) $$\begin{array}{c} {\text{obj}}^{*}=-\frac{1}{2}\sum_{j=1}^{\gamma }\frac{G_{j}}{H_{j}+\lambda }. \end{array}$$

The sample data are divided based on the objective function. We choose features for the training set using the split sample data, train the model using a portion of the chosen features, and then assess the test set using the same feature scheme [30, 31].

One of the highlights of XGBoost is the definition of a splitting criterion that maximizes the reduction in loss at each optimal splitting point. This is one of the reasons for the efficiency of XGBoost, where the gain is defined by subtracting the pre-split structural score from the post-split structural score and choosing the split point with the greatest gain as the optimal split point, in the sense of the split point that results in the greatest reduction in model loss compared with the pre-split loss. Such a gain definition method fits the residual tree of the round very well. Therefore, we chose the XGBoost algorithm to further evaluate the exploration of the pathway of civic education in higher education.

### 3.2. Investigating the Primary Political and Ideological Education Routes within the Framework of Big Data

Deep big data integration with the sphere of political and ideological education is an unavoidable tendency in the current reform and innovation of education. University students, as a group with an active mind and a high level of network utilization, are also the primary venue for schools to carry out network surveillance and network propaganda [32]. The school's education model and educational philosophy and way of thinking will be impacted by the wave of big data. In this study, we examine four factors that support innovation and the growth of political and ideological work, such as the development of big data thinking innovation, work method innovation, work carrier innovation, and ideological work team creation [33, 34].  Figure 2 illustrates the steps to explore in enhancing the way universities approach ideological and political education in the era of big data. It is helpful to comprehensively and dynamically grasp and continuously follow up the educational object and plays an important role in improving the effectiveness of ideological and political education in colleges and universities.

#### 3.2.1. Cultivate Big Data Thinking

First and foremost, all university functional departments should adopt the idea of “Big Thinking and Administration” to collaborate, unify, and coordinate, adhere to the idea of “student-oriented” education, and pay special attention to the advancement of platforms for network administration and thinking. The school should coordinate and integrate the data resources of all departments to build a consistent, workable, and efficient data network platform. The development of a big data network information platform that combines data collection, software development, quantitative analysis, data processing, and network warning functions to achieve full staff education, full education, and all-around education should be the responsibility of the network management department. This department should also take the lead in monitoring network public opinion. To improve education effectiveness, thinking and political science professionals should improve data sensitivity, accurately identify data from numerous data centers, including college students' thought dynamics and value orientation, and carry out scientific storage and efficient use of the data in combination with the traditional political and ideological education model.

#### 3.2.2. Innovation in Working Methods

Educators in politics and ideologies should first implement big data technology into their operations to accurately gather, count, and analyze data, quickly identify students' psychological issues and ideological dynamics, and use the big data platform as a carrier to inform the development of work in these fields. To understand student growth trends and conduct targeted student activities, data on student financial aid awards, academic achievement statistics, participation in online ideological activities, and consumption preferences since their enrolling can be collected. Second, a sizable database should be actively used to conduct varied student evaluation. Political and ideological education cannot be carried out by evaluating pupils using uniform criteria or educating them using uniform practices. Third, we need to actively understand the early warning system. The basis of big data technology is forecasting, or the ability to foresee potential events in the future through data analysis. Ideological and political workers can understand the circumstances of ideological fluctuations for some students who have psychological issues and academic challenges through data analysis and then carry out educational counseling and psychological intervention for the corresponding students.

#### 3.2.3. Work Carrier Innovation

Today's college students use self-media as a platform for networking and learning due to the ubiquity of mobile Internet. By grasping students' demands for the Internet and following up on the era of big data, more new activities are created to proactively occupy the position of online ideological and political education. The use of online videos and new media platforms is to strengthen patriotism education and ideological and political education, and actively spread social energy. To further reduce the gap between teachers and pupils, the majority of ideological and political workers and educators should take the effort to master the new network language and actively engage with the education goal. To improve the coherence and appeal of online ideological and political education in a way that is nice and acceptable to university students, students can experience an ideological baptism in a peaceful process, sort out their academic confusion, and declare their growth goals.

#### 3.2.4. Team Building Innovation

The real application of big data technology to realize its scientific and social value involves creating a competent team with a strong sense of accountability inside the network thinking and political sphere. “Big Data” ideological and political education should actively encourage big data thinking, learn how to use big data technology in educational endeavors, master the use of big data, improve insight into the value of data, and combine the knowledge and abilities of traditional ideological and political education work to create an integrated development that combines online and offline learning. Based on this, political and ideological professionals should seek to advance political theory studies, take a strong political position, and improve ideological and political quality in order to assist students develop a proper perspective on life and values. The university's network management division should also actively coordinate training for big data technical staff to address issues with data analysis, supervision, and management. Additionally, it should continuously help ideological and political workers to swiftly and effectively analyze data in accordance with the standards of ease and speed, as well as to build their capacity to perform big data analysis and network ideological and political activity [35].

## 4. Discussion and Analysis of Results

Recently, the times have been concentrating on the organic integration of big data concepts, methodologies, and ideological and political teaching in colleges and institutions. The current challenge is to study the path of ideological and political education from the cultivation of big data thinking innovation, work method innovation, work carrier innovation, ideological work team creation, and other elements using big data technology as the core carrier. As a result, political and ideological teaching in colleges and universities will be more effective in the big data era.

The ability to accurately and effectively use Internet technology to carry out education in politics and ideology activities is another important metric of an ideological and political worker's level of working ability. An accurate understanding of student information and dynamics is the foundation for carrying out ideological and political education work. Access to college students' ideological dynamics, consumption patterns, and range of activities can help educators better understand students' current circumstances, speed up the education preparation process, and help some students understand their families' financial situation, the propensity for psychological issues, and their ideological ideologies.

On the one hand, access to student data will become even more rapid with the arrival of the big data era. On the other hand, it will be possible for the first time to grasp the electronic footprints that students have left in their learning and daily lives, eliminating the flaws of ideological and political workers using traditional data forms statistics, doing away with the laborious process of information gathering, and accelerating the use of data to solve problems. However, big data provide the advantages of comprehensive coverage and efficient accuracy, which reduces unnecessary time loss. It addresses every facet of children's behavior in school. To better understand the recognition and feelings of the students in the aforementioned teaching step, the experimental group's students were evaluated following the teaching experiment using a feedback questionnaire. The outcomes are displayed in Table 1.

Following the teaching experiment, the experimental group's pupils' attitudes were as follows: warmly welcome (65%); welcome (25%); general (6%); very unwelcome (4%); and absolutely not welcome (0%). Overall, this method of instruction is well-liked by students. The learning outcomes of students can be improved, the problem of tedious learning in the traditional classroom can be partially solved, and the teaching in the classroom can be improved using this type of teaching methodology. It can also make ideological and political courses or machine learning interesting for students.  Figure 3 is used to illustrate the change in student opinions as a function of the survey's response rate, which demonstrated the validity and reliability of the survey.

For university students to engage in political and ideological work, thought dynamics are crucial, but the ability to grasp ideological consciousness has the trait of concealment, if the grasp of the students' ideological condition is inaccurate not only makes the educational effect counterproductive but also is not conducive to educators to accurately carry out education in politics and ideology activities. With the increasing diversification of college students' thoughts and learning styles, the traditional means of student work can hardly meet the needs of students' individuality and diversification. Education is a long-term process of continuous consolidation and improvement. Statistics that track data may quickly show pupils' dynamic changes, which is helpful for ideological and political education in tasks such as adjusting, consolidating, and analyzing. Offline instruction with online analysis is combined, the two via a data platform are integrated, and students in actively predicting, modifying, and supervising the ideological and political workers to carry out the ongoing normalization and improvement of the educational effect are engaged.

Big data information statistics are of a long-term and ongoing nature, but the software platforms utilized by universities vary and there are no uniform standards or data collection criteria.  Figure 4 displays the results of the questionnaire we created to gauge how the new teaching method was impacting student learning.

In the current online society, university students are easily influenced by all kinds of online information, and the virtual nature of the online environment can easily lead to self-indulgence in the process of online interactions, detaching them from real-life interactions and activities. Some university students have unhealthy hearts and are under great psychological pressure. The function of education is to train students to become an independent and well-rounded individual, and it is important to awaken the mind and develop a sound personality. Due to the lack of regulation and guidance of the network, the lack of training on the supervisory ability of this network platform for thinking and political work, the irrational interactive environment on the network can cause the variation of democratic participation forms and easily cause group incidents at special time points. Some university students have excessive behavior, improper speech, interpersonal relationship alienation, and other bad phenomena, so the ideological and political education activities are very necessary.

Following their learning experiences with this kind of education, the findings show that 70% of students view it as extremely effective, 20% rate it as effective, and 10% rate it as doubtful. In a nutshell, the use of machine learning in ideological and political course content has stoked students' interest in learning new things and aided in their mastery of both the big data and political and ideological course content. This method of education thereby aids learners in achieving higher course learning results.  Figure 5 demonstrates the relationship between the change in students' learning effect and the number of respondents, demonstrating the validity and reliability of our survey.

As seen in Table 2, we also looked at how much attention students paid to ideological and political courses. The following statistics demonstrate the impact of students' attention on learning in the experimental group: 60% of students thought it was extremely positive, 30% thought it was beneficial, 5% said they were unsure, and 5% believed it was unfavorable. As a result, the majority of students think that the use of machine learning will help them concentrate while also giving them a brief immersion experience. Students who are aware of their disadvantage might grow weary after a long study session and temporarily lose interest in what they are learning. Naturally, there is a problem with the human intellect here. In conclusion, big data education is crucial for improving students' attention spans.  Figure 6 shows how students' attention changed as the number of respondents changed, demonstrating the survey's validity and reliability.

According to the aforementioned poll, A, B, C, and D, respectively, indicate “fostering big data thinking innovation, working technique innovation, work carrier innovation, and ideological work team formation.” Figure 7 illustrates how the XGBoost algorithm is used to rank and assess the importance of each test variable to the creation of political and ideological education curricula in higher education institutions.

Based on the above survey, we further analyze the importance of fostering innovation in big data thinking, innovation in working methods, innovation in working carriers, and construction of ideological work teams in exploring thinking education. We used the XGBoost algorithm to select the features in the questionnaire, trained the model with the selected subset of features, and then evaluated the four innovation paths under the same feature scheme. The membership variables of “cultivating big data thinking innovation, work method innovation, work carrier innovation, and ideological work team building” are denoted by A, B, C, and D, respectively.

The XGBoost algorithm was used to rank and analyze the importance of the variables explored in the pathway of enhancing political education in higher education, and Figure 7 shows the results of the importance ranking for each variable. In general, the importance score measures the value of the feature in the construction of the enhancement decision tree in the model. The more an attribute is used to build a decision tree in the model, the higher its relative importance. Attribute importance is obtained by calculating and ranking each attribute in the dataset. Attribute importance is calculated by the amount of each attribute split point improvement performance measure in a single decision number, with the node responsible for weighting and recording the number of times. This means that the larger the attribute's contribution to the split point improvement performance measure, the greater the weight; the more boosted trees it is selected by, the more important the attribute is. Ultimately, the results of an attribute in all boosting trees are weighted and summed and then averaged to obtain an importance score.

The experimental results indicate that consideration of work-related innovation comes in last and that the evolution of big data concepts as the second-most crucial strategy to enhance political and ideological instruction in colleges and universities is innovation. Based on this, ideological and political workers should monitor student involvement and communication on the Internet platform and promptly modify instructional strategies and technical tools. At the same time, universities should also place a high value to this platform of network thinking politics to give financial support and material protection, otherwise there will be difficult to promote long-term sustainable situation.

## 5. Conclusions

The introduction of big data and the onset of the era of big data bring about significant changes in how human society thinks about and behaves to change the world. The emergence of big data and the coming of the big data era have brought great changes to the way of thinking of human society in understanding the world and the way of behavior in transforming the world, and the innovative development of ideological and political education in colleges and universities has also presented a situation of both opportunities and challenges. This study investigates and studies the influence of students' attitudes and learning effects on the integration of big data into ideological and political education. Further, it is oriented to study and analyze the dilemmas and challenges facing the ideological and political education in universities in the era of big data and promote the innovative development of ideological and political work in four aspects, such as cultivating innovation in big data thinking, innovation in working methods, innovation in working carriers, and construction of ideological work teams. The experimental results show that the innovation of working methods in the era of big data has a greater role in improving the path of ideological and political education in colleges and universities, and we hope that it will be of some help to the educational work of colleges and universities. Based on this, data analysis and ideological and political education should be combined and thoroughly implemented in all stages of ideological and political education to improve the overall quality and moral quality of college students, comprehensively improve the work efficiency of university ideological and political work, and cultivate more high-quality talents for the country.

In the context of the era of big data, networking and datafication have become an important driving force for educational reform and innovative ways of educating people. Therefore, we must continue to innovate the concept of ideological and political education for nurturing people and management mode and cultivate composite and innovative talents in the context of the new era. The advent of the era of big data has brought challenges to traditional ideological and political education, but it is also an important opportunity for the majority of ideological and political workers to make good use of the Internet platform to expand the path of education and to promote the modernization of network ideology.

## Figures and Tables

**Figure 1:** Working principle of the XGBoost algorithm.

**Figure 2:** Ideas for improving the way that colleges think and educate in the big data era.

**Figure 3:** Change in students' attitudes with the number of respondents.

**Figure 4:** Impact of big data on students' political and ideological education.

**Figure 5:** Changes in students' learning effect with the number of respondents.

**Figure 6:** Changes in students' attention with the number of respondents.

**Figure 7:** Importance ranking of four working path features.

**Table 1:** Big data attitudes among students are interwoven with their political and ideological education.

Attitude	Warmly welcome	Welcome	General	Very unwelcome	Absolutely not welcome
Percentage	65	25	6	4	0

**Table 2:** Big data's impact on pupils' learning abilities when combined with ideological and political instruction.

Influence	Very vigorous	Vigorous	Not sure	Inactive	Very inactive
Percentage	60	30	5	5	0

## Data Availability

The authors declare that the research was conducted in the absence of any commercial or financial relationships that could be construed as potential conflicts of interest.
